# College Student Social Dynamic Analysis and Educational Mechanism Using Big Data Technology

**DOI:** 10.1155/2022/7132817

**Published:** 2022-07-05

**Authors:** Jing Bai

**Affiliations:** Zhengzhou Preschool Education College, Zhengzhou 450000, China

## Abstract

With the advancement of the “big data” technology, college students inadvertently purchase personal advice while taking advantage of the exciting Internet to access information quickly and easily. In order to objectively achieve the real office of college students' material enlightenment penetration in the mobile-friendly network, we choose the popular mobile social network, and we apply the natural clustering algorithm rules to segment the college students. Further, we identify college students, based on which we construct information leakage and apply the risk assessment design. The comprehensive entrepreneurial evaluation of the microblog platform combined with the user's mobile complaints is utilized to conduct a psychological analysis on the key components and key communication channels of college students' complaint leakage. We obtain ticket data using the social prospect method and refer to four dogmatic characteristic elements of query motivation. And we also collect dimensions through surrogate analysis. Based on the reference feature factor, four different user groups are rapidly moved. Dining, social, teaching and large users, and the model features of various usage profiles are described in combination with eight categories of user feature importance. The |objective is to improve college students' awareness of social network and mobile partner network mobile information to a certain extent. We attempt to protect college students from fraud and installation plans, to standardize the management of online social platform of advertisements, and to progressively promote the disposal of network movable property due to security changes.

## 1. Introduction

With the evolution of mobile Internet photography, the amount of all-encompassing data has exploded. People can easily and quickly obtain utilitarian appeals from massive data. And at the same time, netizens' concern for the Internet is deepening. On April 28, 2020, the China Internet Network Information Center (CNNIC) released the 45th “Statistical Report on China's Internet Development.” As of March 2020, the number of netizens in my family has reached 904 million, and the wisdom rate has reached 64.5%. This scale exceeds 897 million, the Internet penetration rate exceeds 60%, and the usage rates of Moments, Weibo, and Qzone are 85.1%, 42.5%, and 47.6%, respectively [1]. Among the apps commonly used by active netizens, instant messaging apps and social apps still occupy an absolute proportion. As a festival media platform and a companion media platform, Weibo is driving constant growth in user usage with the in-depth deployment of sudden videos and mobile live broadcasts and the gradual increase in services. Meanwhile, mesh communication platforms remain the primary way people helping and contacting each other. College students are a special group in mobile social networks. As they step onto a college campus, evoking the unbridled college energy, their sense of independence gradually multiplies. Meanwhile, they have more free tense than in the noble crowd. They use exciting social platforms like WeChat, QQ, and Weibo to enrich their extracurricular life every day. Also, they are already responsible for their personal teaching and even their intimate relationships when they gossip, grab Weibo, and buy updates online. Recalling the days of donkey friends, with the increase of network technology, network atrocities, network rumors, and other incidents, many scholars began to study and think about the leakage of user intimacy in mobile communication networks [2–8]. Tzavela et al. customized an advertisement traceability system and continuously tracked the relief activities of 150 Weibo users. They cited the basic characteristics of users and loneliness instructions for credibility analysis and investigation and obtained the main channels and objects of user opinion leakage [9]; Zhe customized MapReduce technology and backtracked netizen data through joint permissions. They afterwards formulated the personalized secret safety strategies and decomposed the relationship between users' sincere-feature intimity, double-attribute seclusion and several-ascribe intimacy [10]. The authors choose six ideal and unsettled conversible apps. They conducted venture assessment on movable app user privacy escape risk through expert records, supported on which they escort psychological analysis on the use of intimity complaint leakage peril evaluation index system supported on the figure user friendship complaint escape probability valuation index system [11].

Researchers [12] analyzed the accessibility dilemma of college students dropping out in mobile social networks through online questionnaires. They gave a certain degree of protection to the intimate relationship of Zhang and others. The importance analysis of retirement risk concept is constructed using risk perception hypothesis and information privacy concern speculation, wherein the entity agent of college students' mobile festival media privacy hazard cognition is analyzed. Most of these research incidents focus on the intimate protection and access rights of friendly web users publishing gospel or article content. Meanwhile, there are few studies on the disclosure of college students' mobile instructions in the volatile festival web. Some existing reviews mainly preserve the basic data of college students through conference reconnaissance, online questionnaires, and so on. This is conducted without the characteristics of deep thinking about big data, and there is a certain subjectivity. In the context of big data, this paper conducts creep usage instructions in a familiar grid; we use a clustering algorithm to identify college students among them, based on which we analyze the authenticity of usage information and further use cutting-edge escape hazard assessment criteria to escort hazard analysis. In summary, our model is built upon the factors of college students' text message leaking keyboard and targeted preventive measures.

In this work, the authors have tilted the way of college students' festival network mainly from the following aspects: the influence of festival network customs on social participation, the collision of friendship complex on academician's deeds, and the motivation of college students to accompany online classes. In addition, we established a classification model of college students' holiday mesh action intervention. However, the constructed model needs to be optimized according to the specific situation in order to be accepted by Chinese college students. Herein, we take together, the motivations, effects, and interventions of columns into account, as shown in Figure 1.

## 2. Related Work

College students, as an extraordinary group with a large proportion of excited social networks, are unique in the following ways. First, they have the opportunity to gain free time during college, which allows them to grow on more exciting social networks and time online. Thus, the online time is regular. Second, college students have deep acquaintance and curiosity, and thus, the mobile and friendly social networking sites are the main distance for them to obtain advertisements and get involved in knowledge. They are also the capital distance for their excitement and emotional catharsis and finally, also, the most important parade. Annoyingly, these college students' awareness of mobile information protection and privacy protection is very weak. They virtually register teaching in a joyful grid, freely posting dynamic information including location intelligence and family status intelligence. They are inadvertently revealing to the movable preferences and other separate data. In order to prevent the personal information of college students from being used by criminals, these users need to be identified first.

User persona is a “practical description of real users,” which can classify users into different tags according to their behaviors and motivations. This refers to the common characteristics of various users. This can make corresponding descriptions for factors such as differences, photos, and scenes. Generated using the original [4–7], it generally includes three elements of user attribution, user characteristics, and use tickets. The authors [8] constructed user portraits and built a price system to collect use attribute data. The employment data mining method is used to characterize different features. They refined use characteristics later on. Many scholars collect data through common survey methods such as conferences [3–11], observations, and questionnaires and conduct behavioral profiling checks. For example, Tzavela et al. collected online behavioral data of 72 adolescents through semistructured ad hoc interviews [9]. The question-based approach accumulated applicable data for digital natives and used attractiveness graphs to decline stage characteristics in the use of behavior process. Various typical usage profiles are produced [10] accordingly. Data on psychological preferences and other aspects are leveraged [11]. There are two main ways to use the lineage of features: the nature of the keyboard and the lineage of technology. Manual essence is supported by relevant theories, combined with descriptions and essence usage characteristics of academics and researchers [12]. This corresponds to censorship scenarios with a small amount of data, such as the work in [13], interviews, and combined with expert advice to cite user characteristics [14]. Technical extraction is to degrade user characteristics through machine learning algorithms, which is consistent with the censorship scenario of massive use of data. For example, Lin and Xie used the LDA model to text-mine Weibo topics of interest to users and used the opportunity of using priority topics to assign space vectors to expect users. Similarity enables classification and feature extraction of user families [13]. In the detailed and explicit management of user characteristics, it is necessary to further extract marker information from user characteristics. They expand the use of portraits with various perceptual and obvious visual graphics (such as cue clouds or manifold statistical graphics).

The works [15–22] are mostly based on an analysis of 54 empirical literatures that have been informed of censorship by online users of festivals. There are five requirements to understand the needs of “online partners,” namely, cognitive needs, emotional needs, pain withdrawal needs, physical integration needs, and social integration needs. The framework of the influencing factors of social network user behavior consists of 31 particular and inevitable 5 categories, which more comprehensively open up the behavioral motivation of familiar Internet users. The inevitable meanings of these five categories are as follows: cognitive inevitability (8 items), needs related to satisfying physical curiosity or desire for insight; affective needs (5 special needs), indispensable for sharing emotion, pleasure, feeling, and aesthetics; essential integration (8 cues), with hoax-revere, trustworthiness, personification-confidence, stability-related, and state-related; communicative integration needs (7 items), need to be told to connect with family, approvers, and family members. Nowadays, press release is required (3 items), needs to be reported to Sally and Entertainment tells.

## 3. Our Proposed Method

Identify other content that satisfies the delineation that ends each subcluster; building a category system is the condition and basis for collecting data and clearly labeling the unique characteristics of each component. Among the methods to accurately identify the demand motivation of college students' social network travel, the central group processing method helps to standardize the relevant labels of demand motivation arrival. This standard is determined by

(1) $$\begin{array}{c} SA\left(u_{1},u_{2}\right)=\frac{\alpha \beta \left|at-H\left(x\right)\right|}{\left|A\right|}. \end{array}$$

Anhui University invited 8 college students who often use familiar mesh sheets and are good at expressing and 2 researchers who were festive nets as members of the centralized assembly therapy and designated a classmate for the whole process of registration. Prior to the discussion, key materials from the Framework for Influencing Factors of Social Network User Behavior were distributed to panelists. The group discussion was divided into three rounds: the first round disseminated the rationality of the 31 precise requirements in the “Framework of Social Network User Behavior Influencing Factors” one by one. and its applicability in college students; the second round fully discusses the insufficiency of query demand in the “Framework of Social Network User Behavior Influencing Factors”; the third round determines the latest demand drivers and their significance. After three rounds of discussion, delete “opportunity” (unclear meaning), “practical/purpose” (unknown meaning), “indispensable feast” (unclear meaning), “emotional needs” (illogical setting), “accompanying” (unclear meaning), “personal integration needs” (oversetting), “overexpression” (belonging to embody-vent), “creativity” (belonging to ambiguous connotation), “coordination” (belonging to association), “blood connection” “(belonging to confirmation relationship), and other 10 needs; change “control” to “influence others,” change “communication needs” to “communication”; increase “commercial promotion.” Finally, 22 categories of demand motivation areas were formed. This is calculated as

(2) $$\begin{array}{c} J=\overset{k}{\underset{i=1}{\sum }}\overset{W}{\underset{j=1}{\sum }}S\left(x_{j},c\_i\right). \end{array}$$

In order to show the social network behavior characteristics of college students, the demographic attributes and bearing attribution are employed as the pacification reach of college students' familiar network act characteristics; among them, the demographic characteristics include gender, college, earnestness, adult, celebrity, and graduate, which revert the college students' social fret manners. The resource dimension and behavioral attributes include crowd and longitude, which are perceived as college-friendly mesh bearing strengths. Therefore, the behavioral labeling system of college students' social network includes three dimensions: demographic characteristics, behavioral reputation, and problem needs. The questionnaire consists of 30 questions, of which 8 points are used for the characteristic dimension, and 22 debates are used to measure motivation and needs; the numerical level from small to large in the Likert 5 scale is used to infer the value cognition level of college students in the process of online communication behavior. After the sketch of the questionnaire was completed, 15 teachers and students (5 teachers and 10 students) of Anhui University were asked to fill out the questionnaire. According to the results of the Larsen effect, some sentence descriptions are modified to form a rigid questionnaire. Data were obtained through a coalition of paper questionnaires and online surveys from April 2019 to June 2019. The virtual survey recovered 280 valid questionnaires, and the online survey recovered 297 valid questionnaires. We access to complete 577 strong questionnaires. The reliability of the 22 local scales of the motivation dimension is experimental, and the Cronbach alpha cooperation coefficient of the 22 items is 0.921 (>0.7), indicating that the reliability of the questionnaire is high; the range is between 0.915 and 0.922, and the questionnaire is repeated The consistency of the measurement is high, and there is no need to omit the step details. Then, SPSS was used to test the validity of the 22 scale items of the demand motivation dimension, and the KMO import was 0.926 (>0.900), corresponding to factor analysis. This observation is calculated as

(3) $$\begin{array}{c} \text{sig}\left(a,A,D\right)=\frac{\text{Po}{\text{s}}_{\lambda }\left(D\right)-\text{Po}{\text{s}}_{A-\lambda }\left(D\right)}{\left|U\right|}. \end{array}$$

In fashion fitted to the characteristics of differentiated custom patterns, 22 variables of query motivation are used as dimensional guide to obtain their appearance constituent. In SPSS, the descent element of “Cause Integral System” and “Limited Variance Rotation Method” is Embarrass, the parentage tenet is adapted as secret importance better than 1, and the whole controversy and the air sloppy plat are explicate)get.) and a body of rotated elements. As shown, the unmeasured item's loading value for both agents is greater than 0.45 at the same measurement, and the cargo appreciation for each measurement item is greater than 0.45 by an unquestioned factor [16], so there is no poverty-removal measurement hint. The four categorical feature substitutions are high according to each mapped factor loading luminance. Feature replacement 1: this feature component is described as seeking conditions, self-exclusion, incentive compensation, gaining recognition, restraining others, recording specificity, business promotion, etc. It embodies the tendency of college students to apply social networks to present themselves, cut information, etc. and is named cleave, exhibit. Characteristic factor 2: this characteristic factor is informed of information search, information sharing, understanding/observation, friendly supervision, knowledge acquisition, problem solving, etc. It reflects college students' perceptions of the importance of safety-related instruction or awareness from friendly networks and is fully valued, for intelligence acquisition. Characteristic factor 3: the representative agent is related to the company, maintains relationships, and tries new relationships, social bridges, etc., which embodies the requirements of college students for the wearable switchable plexus to specify connections with others and society, collectively referred to as social interaction. Trait 4: this trait is described as execute/flight, escapism, charming age, relaxed self, driven by precision, etc. It reflects that college students like to entertain themselves and release their impressions with joyful troubles, and it is characteristic, entertaining, and relaxing.

Most of the current research on privacy penetration hazard assessment is based on the BS 7799 (ISO/IEC17799) evaluation criterion ethics, and reciprocity indicators are selected from the dimensions of volatile terminals, volatile neural plexus environments, and users themselves. This fiction is mainly based on the vacancy of the user's own subjective dimension and studies the situation of college students' intentional or unintentional disclosure of personal privacy information when recording, logging in, and divulging instructions. Since there are many attributes of attribution barriers used in university research and each attribute has a different impact on the leakage of personal complaints, it cannot be integrated in the analysis, but it is inevitable to exclude attributes with higher attribution importance for analysis. According to the description of the importance of reputation 4, this wallpaper preliminarily calculates the importance of each reputation and selects 14 betting indicators that privately tell the privacy of chattels, as shown in Table 1. Define 4 feature master degrees. Let *W*_*S*_ be the microblog system, and *α*_a_ represents the attribute significance of each risk arrow used, which is determined as

(4) $$\begin{array}{c} \alpha_{\text{a}}=\text{POS }A\left(D\right)-\text{POS}\left(A-\left\{a\right\}\right)\left(D\right)\left|U\right|. \end{array}$$

Among them, *a* is the reputation in the use of reputation adjustment, that is, *a* ∈ *A*; the consequences of using each attribution can be expressed as {*a*1, *a*2, ⋯, *a*|*A*|}, *a* ∈ [0, 1]; *D* is the decision attribute in reputation determination *A*.

## 4. Experimental Results and Analysis

After four different shape factors, all samples were clustered to terminate the mob counts of behavioral portraits. There are 577 observations in this muse, and it is suitable to select the *K*-means algorithm rule to perform cluster analysis on the four eigenfactors in the alternative analysis results. In empirical applications using segmentation, it is more appropriate to limit the scalar of clusters to 4-7 categories [17], so this thinking indicates the fast crowd as 4-7 categories, as shown in Table 1. When the clusters are 5, 6, and 7, the variance of the *F* values of the four canonical components in the ANOVA summary is small, indicating that the differences between the behavioral profiles are not positive; when the cluster is 4, the differences in the *F* values are corrected. Therefore, the scalar for crowd is determined to be 4.

When there are 4 clusters, the closure number and crowd kernel utility of various portraits on each feature component are shown in Table 2, and the single-highway ANOVA process for group and feature proxy variables is shown in Table 2. From the data in Tables 1 and 2, it can be seen that each token of the user has a clear difference in each feature element. The first category of users has the largest crowd-centered rating and restricted hospitality and leisure characteristics, depicting the meridian sense of entertainment value and unemployment in the familiar mesh structure of such users, a symbol of such users known as feast stamps. The second type of users has the largest group center value and import volume in the expression of social communication characteristics, indicating that this type of user has the meridian awareness imported from social network festival communication, and this type of user is a symbol of friendliness. The third user logo is in the information. The acquired feature words have the largest cluster focus value and mean value, indicating that the user instance has the meridian value cognition familiar with network intelligence acquisition, and the user is marked as information style. The quarterly user group's group core effectiveness and excellent quality in social networking, intelligent access, distribution and display, banquet and leisure, etc. remained high, indicating that this user group has a high understanding of the value of social networks in all aspects. It is said to be comprehensive.

In order to show the changeable usage profiles obtained by the above cluster analysis, the cases clustered as 1, 2, 3, and 4 are deducted as modern data tables in SPSS. First, a psychoanalysis of the imposed motivation dimension was performed using the wordcloud2 package in R idiom. The 22 tags are relatively drawn into the attachment cloud, and then, realistic statistical analysis is performed on the 8 tags of the user feature dimension of these 4 types of user portraits. Since the number of people corresponding to each label is different, in order to obtain the consistency of the dimension of the characteristics of each label of similarity, the percentage of the number of users representing the symbol to the total number of labels is used as the load, as shown in Table 2.

The demand motivation dimensions are as follows: amusement, escapism, and being precisely driven are the essential motivations of leisure college students. For the importance of user characteristics, 17% of boys and 8% of girls belong to this category, and the lot of boys is significantly higher than that of girls; 16% of Anhui students, 11% of Jiangsu students, and 9% of Guizhou students belong to this category, Anhui. The proportion of students is much higher than that of girls. 17% of the major electronic computer leagues belong to this category, the largest number of places; 22% of the students in the bottom 30% belong to this kingdom, and only 9% of the students in the top 30% belong to this category; 20% of students belong to this category, while only 3% of casual students fall into this category; grade distribution, celebrity quality distribution, and dates of use are fairly even. According to the above description, the typical characteristics of leisure college students are taken as the criterion, as shown in Table 2.

Demand motivation and demand scale are as follows: maintaining relationships, communication, festival bridges, etc. are the key motivations for social college students. In the user characteristic dimension, 26% of boys and 28% of girls belong to this category, and the proportion of girls is slightly higher than that of boys; 35% of Jiangsu students, 28% of Anhui students, and 21% of Guizhou students belong to this department, and Jiangsu students are much higher than boys. 31% of gay college students and above belong to this category, with the largest symmetry; 31% of computer major leagues belong to this tribe, with the largest quota; 34% of serious star students belong to this category, with the largest proportion; the top 30% of the students fall into this category, with the largest share; 30% of students with frequent habits belong to this order, with the largest share; 32% of students who use 2-3 hours of age belong to this tribe, the largest in scale. According to the above description, the metaphorical characteristics of social college students are obtained. Demand motivation measurements are as follows: social supervision, instruction search, information dividends, etc. are the key motivations of users of the School of Information. In the user-specific proportion, 29% of boys and 25% of girls belong to this family, and the proportion of boys is slightly higher than that of girls; 38% of Guizhou students, 28% of Anhui students, and 8% of Jiangsu students belong to this order; the proportion of Guizhou students is obvious. 35% of sophomores die in this group, the largest quota; 31% of biology majors fall into this group, the largest share; 31% of students in the top 30%-50% change sink into this kingdom, the largest share; 59% of students who apply occasionally fall into this predicament and on a much larger scale; 60% of students who use less than 1 hour at a time belong to this family and on a larger scale; distribution of character traits is relatively uniform.

## 5. Conclusions

In this paper, the method of social survey is used to obtain the label data of college students, and four classification characteristic factors are extracted through factor analysis. Based on the classification of user portraits of groups, the key features of four types of user portraits are analyzed and described in combination with the eight labels of the user feature dimension. Due to limited energy, this survey is limited to three provinces of Anhui, Jiangsu, and Guizhou. At the same time, the characteristics of social network behavior of college students at different levels of colleges and universities are not distinguished. In future research, the survey area and types of colleges will be expanded, and the survey data will be gradually enriched. At the same time, we will explore more statistically significant feature description methods in order to conduct more scientific and in-depth research on college students' social network behavior.

## Figures and Tables

**Figure 1:** An illustration of social media platform for enhancing the education of college students.

**Table 1:** Cluster center and the number of examples.

Cate. #	Cate 1	Cate 2	Cate 3	Cate 4
Sharing	-0.02	-0.31	-0.21	0.83
Info. Ac	-1.23	0.43	0.04	0.37
Comm.	-0.08	0.73	0.32	0.24
Enter.	0.93	-0.16	0.17	0.12
Example #	72	153	132	163

**Table 2:** Category and attribute factor analysis.

Factor	Category	Average	Group F	Factor	Category	Average	Group F
Sharing display	1	3.221	213.334	Communication skills	1	3.432	174.446
	2	2.565			2	2.443	
	3	3.656			3	4.390	
	4	4.354			4	3.435	
Information acquisition	1	2.321	104.556	Entertainment	1	2.435	71.231
	2	3.442			2	3.443	
	3	5. 465			3	2.546	
	4	2.324			4	4.337	

## Data Availability

The data used to support the findings of this study are available from the corresponding author upon request.
